The article "The Fertility Status of the Married People Living with HIV/AIDS in China" was retracted in 2023. Reasons: signs of a paper mill; suspected computer-generated content; unreliable results or conclusions; lack of ethics approval or compliance.

# The Fertility Status of the Married People Living with HIV/AIDS in China

**DOI:** 10.1155/2022/2938340

**Published:** 2022-09-27

**Authors:** Min Que, Guo-ping Ji, Jie Du, Tao Li

**Affiliations:** ^1^Anhui Provincial Center for Woman and Child Health, Hefei 230061, China; ^2^The First Affiliated Hospital, University of Science and Technology of China (Anhui Provincial Hospital), Hefei 230061, China

## Abstract

In order to analyze the fertility status of the married people living with human immunodeficiency virus (HIV)/acquired immune deficiency syndrome (AIDS) (PLHA) of reproductive age in China, a sample of married PLHAs aged 22–45 in China is selected by using a stratified cluster sampling method. All participants are face-to-face interviewed with a structured questionnaire. Among them, the fertility status and its influencing factors of 366 PLHAs are statistically analyzed. Experimental results show that married PLHA of reproductive age in China has a high proportion of having children. The fertility status and fertility intention of females are higher than that of males. The proportion of unwanted pregnancies after the HIV + diagnosis of females is high.

## 1. Introduction

Human immunodeficiency virus (HIV) infection causes acquired immune deficiency syndrome (AIDS), which is one of the most devastating infectious diseases in human history. Although access to the antiretroviral therapy has increased and the number of people newly infected with HIV has continued to decline globally, the incidence, mortality, and new HIV infection rates of HIV/AIDS in China are increasing year-by-year [1]. The infection rate is the highest in middle-aged person, the same-sex transmission has increased notoriously [2], and there are significant regional differences in the prevalence rate [3]. Some key populations have low awareness of HIV, condom use, HIV testing and other health knowledge, and low willingness to test [4]. With the widespread availability of the effective antiretroviral therapy, HIV infection has become a chronic disease, and people living with HIV/AIDS (PLHA) have increased life expectancy [5].

In order to understand the status quo of marriage and childbearing at childbearing age in China, willingness to marry and childbearing and related factors, the project “Research on marriage and childbearing status and willingness to marry and childbearing of HIV-infected persons/patients of childbearing age in China” is carried out from November 2019 to February 2020. This paper uses the fertility-related information of the married PLHA population to analyze the fertility status of the married PLHA population, explore the relevant factors of whether the PLHA population is fertile, and further prevent HIV transmission.

The rest of this paper is organized as follows: Section 2 discusses related work, followed by focusing on statistical methods and related definitions in Section 3. The pregnancy of PLHA and status of existing children are discussed in Section 4.  Section 5 concludes the paper with summary.

## 2. Related Work

After marriage, with the increase of age, all aspects are relatively stable, and with a certain economic foundation, the demand and behavior of having children would increase accordingly. Other studies at home and abroad suggested that the PLHA population without children was more willing to have children than those who had children [6]. It was close to the PLHA population of childbearing age in other parts of China [7] and was not much different from the general population [8]. Interventions must be strengthened to increase the encouragement of HIV-infected women to use contraception in Togo [9]. Although the awareness rate of HIV transmission prevention knowledge and the autonomy of sexual behavior protection among the PLHA population in my country have increased [10], they were affected by the demographic characteristics and related knowledge in different regions [11]. If you had multiple sexual partners for a long time, the proportion of meeting contraceptive needs was not high, which would increase the risk of sexual partners contracting HIV [12].

The research suggested that the PLHA population with low education level in South Florida had a stronger fertility desire and pays more attention to family expectations [13]. The study showed that most PLHAs and their partners had the same desire to have children [14]. Couples considered their own and their spouse's health and marital satisfaction when making reproductive decisions [15]. Preexposure prophylaxis, male circumcision, and ovulation monitoring could effectively reduce the spouse's risk of condom-free sex and HIV infection during pregnancy [16], and medically assisted reproductive technology could be used when it is necessary to reduce the risk of the partner and HIV infection. It increased the conception rate while reducing the risk of offspring transmission, and bred the next generation safely and healthily.

## 3. Statistical Methods and Related Definitions

From the project database of “Research on the Marital Status and Marital Intention of HIV-infected Persons/Patients of Reproductive Age in China,” the general demographic characteristics, fertility, and those who wish to have children are extracted to generate a fertility information database. The project “Research on Marital Status and Marital Intention of HIV-infected/patients of childbearing age in China” adopts the method of stratified cluster sampling, selects 1 city in southern, central, and northern China, and selects 1 to 3 HIV-infected/fertile-age patient cities with a high number of patients. In this study, a face-to-face interview questionnaire is conducted among married PLHAs aged 22–45 in the county (district), and a total of 366 valid questionnaires are obtained.

Statistical analysis is performed with SPSS 22 software. The enumeration data are analyzed by the chi-square test, and the measurement data are analyzed by the variance analysis and independent sample *t*-test. Univariate and multivariate analyses are performed by binary logistic regression analysis, and conditional backwards is used in multivariate logistic regression analysis. The inspection level is *α* = 0.05.

Married in this paper includes a collective term for marital status such as currently married, divorced, and widowed.

## 4. Pregnancy of PLHA and Status of Existing Children

### 4.1. General Demographic Characteristics

The survey subjects are 366 married PLHAs of childbearing age, 275 (75.1%) males, and 91 (24.9%) females, with an average age of (36.19 ± 5.76) years, of which males are 36.27 ± 5.52 years and females are 35.98 ± 6.47 years. 279 persons (76.2%) are married, 76 persons (20.8%) are divorced, and 11 persons (3.0%) are widowed. There are statistically significant differences in age, education level, occupation, personal income, family income, route of infection, and marital status between male and female respondents.

Figure 1 is the general demographic marital status data. It is clearly evident from Figure 1 that there is no statistically significant difference in the distribution of male and female respondents in terms of family size and whether they are only children.

### 4.2. Pregnancy of PLHA Himself or His Spouse

Among the survey respondents, 361 people report pregnancy information of themselves or their spouses, accounting for 98.6%.

Table 1 is the pregnancy status of the married PLHA population of childbearing age in China. It is clearly evident from Table 1 that the number of pregnancies, the number of pregnancies after the diagnosis of HIV infection (HIV+), the number of unintended pregnancies after the diagnosis of HIV+, and the number of live births after the diagnosis of HIV+ are higher than those of male spouses, and the differences are statistically significant (*P* < 0.05).

### 4.3. The Status of Existing Children

323 people have given birth or are willing to give birth in this survey, accounting for 88.3%. The proportions of no child, one child, and two or more children are 18.3%, 46.7%, and 35.0%, respectively.  Table 2 is the status of existing children of married PLHA population of childbearing age in China. It is clearly evident from Table 2 that there is no significant difference in the number of children and the type of children (*P* < 0.05), but the proportion of women who have given birth/willing to have children (94.5%) is much higher than that of men (86.2%), and the difference is statistically significant (*P* < 0.05).

### 4.4. Fertility Desire

Among the 366 married PLHA population, 68 people have the intention to give birth/rebirth, accounting for 18.6%, and 298 people have no intention to give birth/rebirth, accounting for 81.4%.

Figure 2 is the contrast of fertility/rebirth willingness. It is clearly evident from Figure 2 that among the 68 people with the willingness to have children/regeneration, 35.8% (24/68) are without the willingness to bear children, which is higher than 14.7% (44/299) with the willingness to bear children, and the difference is statistically significant (*χ*^2^ = 16.117,).

Figure 3 is the main reasons for willingness to give birth/rebirth. It is clearly evident from Figure 3 that among the 9 reasons why the 68 respondents are willing to give birth/rebirth, the main reasons for choosing the top four are wanting healthy children (50.0%), increasing family fun (48.5%), and wanting to become parents (39.7%).

Figure 4 is the main reasons for unwillingness to have children/rebirth. It is clearly evident from Figure 4 that among the 9 reasons why the 298 respondents do not want to give birth/rebirth, the main reasons for choosing the top three are having children(48.7%), fear of children getting sick (40.6%), and heavy economic burden (38.9%).

### 4.5. Factors Related to Having Children

The related factors of whether 366 respondents have children are analyzed. Taking having children as the dependent variable (having children = 1, having no children = 0), covariates include gender, age, education level, occupation, only child, personal annual income, family annual income, housing situation, marital status, and infection pathway, years of diagnosis, and whether or not to treat. Univariate binary logistic regression analysis finds that, except for gender, infection route, years of diagnosis, and whether or not to treat, other indicators are related to whether there are children (*P* < 0.05).  Table 3 is the analysis of factors related to whether there are children in the married PLHA population of childbearing age in China. It is clearly evident from Table 3 that multivariate binary logistic regression analysis finds that age, educational level, and marital status are all related to whether or not to have children (*P* < 0.05). Univariate and multivariate analysis do not find that gender, route of infection, years of diagnosis, and treatment are associated with having children (*P* > 0.05).

## 5. Conclusion

With the continuous increase in the number of PLHAs in China, the desire of the PLHA population to have children may have a significant impact on public health, and the fertility willingness and behavior of the PLHA population will also be affected by more and more attention. In China, 81.7% of married women of childbearing age have children, 53.2% have two or more pregnancies, and 36.6% had two or more live births. The proportion of women who have had children/willing to have children is higher than that of men. Unintended pregnancy after HIV-positive diagnosis among married women accounts for 28.6%. The related factors of whether married women have children mainly include age, marital status, and education level. The main reasons for fertility/regeneration intention include wanting healthy children, increasing family fun, desire to be a parent, and strong parental expectations. For PLHAs with a strong desire to give birth, they should pay attention to the health service support in key links, carry out necessary health education and counseling, further optimize treatment plans, prevent HIV transmission, and promote maternal and child health, so that more PLHAs can responsibly and freely decide on fertility issues.

## Figures and Tables

**Figure 1:** General demographic marital status data.

**Figure 2:** The contrast of fertility/rebirth willingness.

**Figure 3:** The main reasons for willingness to give birth/rebirth.

**Figure 4:** The main reasons for unwillingness to have children/rebirth.

**Table 1:** Pregnancy status of the married PLHA population of childbearing age in China.

	Males (*n*1 = 270)		Females (*n*2 = 91)		Total (*n* = 361)		*χ * ^2^	*P*
	The number of people	%	The number of people	%	The number of people	%		
The number of pregnancies							6.905	0.032
0	45	16.7	7	7.7	52	14.4		
1	91	33.7	26	28.6	110	32.4		
2 and above	134	49.6	58	63.7	192	53.2		

Live births							2.625	0.269
0	54	20.0	13	14.3	67	18.6		
1	123	45.6	39	42.9	162	44.9		
2 and above	93	34.4	39	42.9	132	36.6		

The number of pregnancies after HIV + diagnosis							18.870	<0.001
0	217	80.4	54	59.3	271	75.1		
1	43	15.9	25	27.5	68	18.8		
2 and above	10	3.7	12	13.2	22	6.1		

The number of unintended pregnancies after HIV + diagnosis							22.970	<0.001
0	247	91.5	65	71.4	312	86.4		
1	18	6.7	15	16.5	33	9.1		
2 and above	5	1.9	11	12.1	16	4.4		

The number of live births after HIV + diagnosis							15.946	<0.001
0	241	89.3	65	71.4	306	84.8		
1	26	9.6	21	23.1	47	13.0		
2 and above	3	1.1	5	5.5	8	2.2		

**Table 2:** The status of existing children of married PLHA population of childbearing age in China.

	Maless (*n*1 = 270)		Female (*n*2 = 91)		Total (*n* = 361)		*χ * ^2^	*P*
	The number of people	%	The number of people	%	The number of people	%		
The number of children							2.862	0.239
No children	54	19.6	13	14.3	67	18.3		
1	131	47.6	40	44.0	171	46.7		
2 or more	90	32.7	38	41.8	128	35.0		

Types of children							2.956	0.399
No children	54	19.6	13	14.3	67	18.3		
Only boys	98	35.6	29	31.9	127	34.7		
Only girls	64	23.3	23	25.3	87	23.8		
Both boys and girls	59	21.5	26	28.6	85	23.2		

Having given birth/willing to have a child							4.569	0.033
No children	38	13.8	5	5.5	43	11.7		
Have children	237	86.2	86	94.5	323	88.3		

**Table 3:** The analysis of factors related to whether there are children in the married PLHA population of childbearing age in China.

Settings	No children (*n*1 = 67)		Having kids (*n*2 = 299)		Univariate		Analysis results	
	The number of people	%	The number of people	%	cOR	*P*	aOR	*P*
Age								
22–29	14	20.9	45	15.1	1		1	
30–39	46	68.7	131	43.8	0.886	0.730	1.331	0.451
40–45	7	10.4	123	41.1	5.467	0.001	5.664	0.001

Educational level								
Junior high school and below	27	40.3	217	72.6	1		1	
High school and above	40	59.7	82	27.4	0.255	<0.001	0.352	0.001

Profession								
Peasant, migrant worker, housework, and others	23	34.3	167	55.9	1			
Business service and business unit	26	38.8	62	20.7	0.328	0.001		
Self-employed and unemployed students	18	26.9	70	23.4	0.536	0.001		

Only child								
No	55	82.1	274	91.6	0.418	0.022		
Yes	12	17.9	25	8.4	4.982	<0.001		

Personal annual income (ten thousand yuan)								
<2	21	31.3	151	50.5	1			
2-	19	28.4	70	23.4	0.512	0.055		
4-	27	40.3	78	26.1	0.402	0.005		

Annual household income (ten thousand yuan)								
<5	27	40.3	180	60.2	1			
5-	21	31.3	80	26.8	0.571	0.081		
10-	19	28.4	39	13.0	0.308	0.001		

Housing situation								
Buy a house	34	50.7	77	25.8	1			
Self-built	21	31.3	162	54.2	3.406	<0.001		
Rent or dormitory	12	17.9	60	20.1	2.208	0.036		

Marital status								
Divorced + widowed	31	46.3	56	18.7	1		1	
Married	36	53.7	243	81.3	22.910	<0.001	4.047	<0.001

## Data Availability

The simulation experiment data used to support the findings of this study are available from the corresponding author upon request.

## References

[1] Qiao Y. c., Xu Y., Jiang D. x. (2019). Epidemiological analyses of regional and age differences of HIV/AIDS prevalence in China, 2004–2016. *International Journal of Infectious Diseases*.

[2] Du M., Yan W., Jing W. (2022). Increasing incidence rates of sexually transmitted infections from 2010 to 2019: an analysis of temporal trends by geographical regions and age groups from the 2019 Global Burden of Disease Study. *BMC Infectious Diseases*.

[3] Leung M. F., Wang J. (2021). Minimax and bi-objective portfolio selection based on collaborative neurodynamic optimization. *IEEE Transactions on Neural Networks and Learning Systems*.

[4] Jiang R., Xin Y., Chen Z., Zhang Y. (2022). A medical big data access control model based on fuzzy trust prediction and regression analysis. *Applied Soft Computing*.

[5] Stiles M. K., Wilde A. A. M., Abrams D. J. (2020). 2020 APHRS/HRS expert consensus statement on the investigation of decedents with sudden unexplained death and patients with sudden cardiac arrest, and of their families. *Heart Rhythm*.

[6] Dubey V. P., Randell K. A., Masonbrink A. R. (2021). Justice system involvement among adolescents in the emergency department. *The Journal of Pediatrics*.

[7] Siegel K., Meunier É., Tocco J. U., Lekas H. M. (2018). Reproductive desires and considerations of HIV-positive men in heterosexual relationships in New York City. *AIDS and Behavior*.

[8] Liu J., Liu M., Zhang S., Ma Q., Wang Q. (2020). Intent to have a second child among Chinese women of childbearing age following China’s new universal two-child policy: a cross-sectional study. *BMJ sexual & reproductive health*.

[9] Yaya I., Patassi A. A., Landoh D. E. (2018). Modern contraceptive use among HIV-infected women attending HIV care centres in Togo: a cross-sectional study. *BMJ Open*.

[10] Gu L. Y., Zhang N., Mayer K. H. (2021). Autonomy-supportive healthcare climate and HIV-related stigma predict linkage to HIV care in men who have sex with men in Ghana, West Africa. *Journal of the International Association of Physicians in AIDS Care*.

[11] Nieuwesteeg B., Faure M. (2018). An analysis of the effectiveness of the EU data breach notification obligation. *Computer Law & Security Report*.

[12] Yu J., Nehl E. J., Dinh V. P. (2020). Vietnamese female sex workers in rural cross-border areas of Guangxi, China: migration and HIV/STI risk behaviors. *AIDS Care*.

[13] Jones D. L., Cook R., Potter J. E. (2016). Fertility desires among women living with HIV. *PLoS One*.

[14] Iliyasu Z., Galadanci H. S., Zubair K. A., Abdullahi H. M., Jalo R. I., Aliyu M. H. (2020). Fertility desire concordance and contraceptive use among couples living with HIV in northern Nigeria. *The European Journal of Contraception and Reproductive Health Care*.

[15] Feyissa T. R., Harris M. L., Loxton D. (2020). They haven’t asked me.I haven’t told them either”: fertility plan discussions between women living with HIV and healthcare providers in western Ethiopia. *Reproductive Health*.

[16] Schwartz S. R., Bassett J., Mutunga L. (2019). HIV incidence, pregnancy, and implementation outcomes from the Sakh’umndeni safer conception project in South Africa: a prospective cohort study. *The lancet HIV*.

